This article has been retracted.

# Network Security Technology of Supply Chain Management Based on Internet of Things and Big Data

**DOI:** 10.1155/2022/7753086

**Published:** 2022-06-21

**Authors:** Xiuchun Lin

**Affiliations:** College of Information and Electrical Engineering, China Agricultural University, Beijing 100083, China

## Abstract

In order to improve the network security of supply chain management based on the Internet of Things and big data, this paper studies the Internet of Things and big data technology and analyzes the data processing process of the Internet of Things. On the premise that the terminal device meets the requirements of delay and energy consumption, a data offloading encryption model is established to offload data to multiple edge servers for encryption. In addition, this paper proposes an optimization problem including overall security, delay, and equipment energy consumption and establishes a mathematical model that maximizes overall security under the condition of satisfying the requirements of delay and equipment energy consumption. From the simulation data, it can be seen that the network security technology of supply chain management based on the Internet of Things and big data proposed in this paper can achieve effective management and control of supply chain nodes and improve their information security.

## 1. Introduction

Since the Internet of Things is an information-sharing network established to serve people and things, it is inevitable that data and privacy will be leaked. Therefore, we need to strengthen the safeguard system in this regard. As a network platform, the Internet of Things is based on big data and cloud sharing, and its development and operation are inseparable from the protection of data and privacy. However, there is currently a lack of unified technology and security legal system, resulting in a lack of sense of security in the Internet of Things. Only on the basis of ensuring network security and privacy security and improving the legal system of security management and guarantee, the Internet of Things can be accepted by more users, and the constraints in development can be lifted, and then the rapid development can be embarked on. This shows that every link in the application of the Internet of Things, such as information collection, aggregation, and transmission determines the security requirements of the Internet of Things.

If there are no effective encryption protection measures in the transmission process of information data, it will lead to the transmission process, whether it is broadcast, multicast, or wireless. The transmitted data may be interrupted midway through interception, deliberate tampering, and other damage. In addition, the heterogeneity and diversity of nodes in the IoT network, endurance, high temperature, and cold resistance, as well as the accuracy and timeliness of information transmission are all related to the security of the network environment and data privacy. Therefore, these all put forward higher requirements for the security protection construction of the Internet of Things.

The Internet of Things needs to rely on various security platforms in running applications such as big data cloud computing and distributed computer systems. It is precisely because of the help of these supporting platforms that promoted the development of the Internet of Things. A safe, reliable, and efficient system must be provided for the upper-layer services and applications of the Internet of Things, which puts forward higher requirements for the security system of the Internet of Things.

It is precisely because of the massive use of sensors in the Internet of Things that the cost of human resources is saved, and some complex and dangerous tasks are performed by humans remotely manipulating machines. In this case, the Internet of Things applications are carried out in the state of unmanned monitoring. In this way, attackers can easily gain access to the internal devices, further, modify and destroy the sensors on the devices, and even illegally manipulate them by deciphering the internal communication protocols. If certain important institutions of the country happen to rely on the Internet of Things, attackers can interfere with the normal operation of the equipment by interfering with the sensors. For example, in the process of long-distance power transmission in the power sector, many substation facilities are remotely controlled through the Internet of Things. Attackers interfere with these devices through illegal operations, and the attackers change the parameters and cause significant impact. The functions of general sensors are simple and easy to be tampered with, which affects their security protection capabilities. Due to the variety of communications involved in the Internet of Things, their data transmission processes do not have specific standards, so they cannot provide a unified security protection system.

In order to improve the network security technology of the supply chain, this paper studies the Internet of Things and big data technology and analyzes the data processing process of the Internet of Things.

## 2. Related Work

Since market competition has been transformed from competition among enterprises to competition among supply chains, effectively managing supply chain risks has become an important part of supply chain competitiveness. People pay more and more attention to the risk management of supply chain. At present, scholars have conducted extensive research on the identification, evaluation, and risk response of traditional supply chain risks. u et al. [1] studied the supply and demand in the supply chain and believed that the suppliers in the supply chain could not supply on time and in quantity due to the lack of productivity or raw materials, and the changes in the demand cycle of consumers in the market led to excessive demand. The phenomenon of too much or too little is supply chain risk, and it is defined as supply risk and demand risk of supply chain, respectively. Ding et al. [2] consider that the appearance of any node in the supply chain will affect the entire supply chain through the study of the mutual influence and interdependence between the nodes of the supply chain. Gu and Liu [3] believe that the “bullwhip effect” in the process of information transmission among enterprises in the supply chain makes the transmitted information distorted and is one of the important sources of supply chain risks. Due to the distortion of information, the enterprises in the supply chain cannot cooperate effectively, resulting in excess inventory costs or out-of-stock losses in the supply chain. When people have a certain awareness and assessment of the risks in the supply chain, they will take some measures to prevent these risks. Chen and Zhao [4] study that if the risk can be discovered in time when the risk invades the supply chain enterprise and corresponding measures can be taken, then the enterprise can avoid the persecution of certain risks. Therefore, the study shows the establishment of a system that can detect the risk when it is intruded through the model. Huang et al. [5] put forward a variety of prevention suggestions on supply chain risks through the research and analysis of supply chain alliance enterprise risks, which clearly points out that effectively coordinating the “three streams” in the supply chain and reducing the unstable links in the supply chain have a negative impact on the supply chain. The prevention of chain risk is of great significance. Yadav et al. [6] analyze supply chain risks through the SCOR model and proposes risk prevention measures. They believe that not only the internal operation of supply chain enterprises can bring risks to the supply chain but also the external environment in which the supply chain is located and the risks in the supply chain. The enterprises in the cooperative relationship can bring corresponding risks to the supply chain. For the abovementioned supply chain risk of information distortion due to the “bullwhip effect,” Tsang et al. [7] empirically analyze the risk management model. In this process, it was found that although preventive risk management of supply chain can reduce the safety stock of enterprises, it cannot alleviate the “bullwhip effect” in supply chain as effectively reactive risk management. At present, the research on the traditional risk and management of the supply chain is relatively detailed and comprehensive, but with the rapid development of the Internet and the application of the Internet in the supply chain, the supply chain has produced many new security risks [8].

Kupriyanovsky et al. [9] identified 9 major network security vulnerabilities based on 92% of the data information in DBIR, including cyber espionage, DOS attack (disk operating system denial of service), crimeware, web application attack, insider abuse, miscellaneous errors, and physical theft. Due to the widespread application of Internet information technology in the supply chain, these network security vulnerabilities have brought a nonnegligible threat to the cyber-physical security of the supply chain [10]. The reason why the supply chain will increasingly rely on Internet communication technology is that it can help the supply chain to achieve efficient information sharing between enterprises, improve the operation efficiency of the supply chain, and reduce the operation cost of the supply chain [11]. Many literature studies have used analytical models and numerical simulations to study and analyze the inventory holding costs and out-of-stock costs saved by enterprises through information sharing through network information technology [12]. Some literature studies also analyze the impact of information sharing on the price structure within the supply chain [13]. There are also many literature studies studying the impact of supply chain information integration. Coatney and Poliak [14] found that the integration and coordination of information in the supply chain can help improve the operational efficiency of the supply chain. Due to the information sharing between supply chain enterprises through Internet information technology, information sharing not only improves the efficiency of the supply chain but also increases the risk of supply network logic security. Since the information shared by enterprises in the supply chain with their partners is relatively important business information, more consideration should be given to the network security of the supply chain when sharing information between enterprises [15].

Kalaivani and Indhumathi [16] clearly pointed out through research that the elasticity construction of supply chain is an important part of supply chain risk management. Alsayaydeh [17] defines the elasticity of supply chain as a kind of enterprise's ability to return to normal under the influence of risk through research and analysis and studies the four factors that affect this elasticity ability including flexibility, speed, visibility, and collaboration aspect. Yan et al. [18] believe that the elasticity of the supply chain emphasizes the ability to respond quickly and recover quickly after encountering risks.

## 3. Data Offload Encryption System Model

The problem studied in this paper is based on the edge computing architecture and considers the data transmission scenario shown in Figure 1. There is a narrowband IoT terminal device and multiple edge servers in the scenario. Moreover, data from end devices are offloaded to multiple edge servers for complex encryption. After encryption is complete, the cipher text and key are transmitted to the cloud server. The system also needs to meet the delay requirements of data transmission and the energy consumption requirements of terminal devices and edge servers.

As shown in Figure 1, the entire system is divided into three layers, namely, one is the device layer, the other is edge layer, and the third is the cloud center layer.

In Figure 1, there is a cloud server that receives data, a terminal device generates data, and K edge servers encrypt the data fragments of the terminal device. Among them, the parameter *a*_*k*,*n*_ indicates that the edge server *k* executes the encryption algorithm *n* and *a*_0,*n*_ indicates that the terminal device executes the encryption algorithm *n*. Among them, there are 8 optional encryption algorithms, and *N*={1,2,…, *n*,…, 8} is used to represent the set of optional encryption algorithms. The parameter *m*_*k*_ represents the data segment distributed to the edge server *k*, *K*={1,2,…, *k*,…, *K*} is used to represent the set of edge servers, and *M*={*m*_1_,…, *m*_*k*_,…, *m*_*K*_} is used to represent the set of data segments obtained by the edge server.

When the terminal device transmits data, data encryption can be used to improve the security. Using encryption algorithm to process terminal data, important data and resources can be transmitted in cipher text, which will not be easily cracked by unauthorized malicious targets. Therefore, the security of data transmission is affected by the encryption algorithm executed by the edge server and the size of the data fragment allocated to the edge server, and how to reasonably quantify the data security is a crucial issue. A security model is introduced to measure the security of edge servers.

When the encryption algorithm runs on different servers, the execution efficiency of the encryption algorithm is different because the CPU speed of the server is different. Here, the efficiency of the encryption algorithm in the multiserver environment is converted. When edge server *k* executes encryption algorithm *n*, the execution efficiency of the converted encryption algorithm is defined as follows:

(1) $$\begin{array}{c} u_{k,n}=\frac{\rho_{n}}{F}\cdot f_{k},\;k=1,2,\ldots ,K;n=1,\ldots ,8, \end{array}$$

(2) $$\begin{array}{c} u_{0,n}=\frac{\rho_{n}}{F}\cdot f_{0},\;n=1,\ldots ,8, \end{array}$$

where *u*_*k*,*n*_ represents the execution efficiency of the encryption algorithm *n* in the edge server *k*, *u*_0,*n*_ represents the execution efficiency of the encryption algorithm *n* in the terminal device, and their changes are determined by the CPU speed *f*_*k*_ of the edge server *k*, *ρ*_*n*_ is the execution efficiency of the encryption algorithm *n* in the literature, F is the CPU speed of the server in the literature, and *f*_0_ is the CPU speed of the terminal device.

The higher the execution efficiency of the encryption algorithm is, the lower the relative complexity and the easier it is to be cracked. According to the execution efficiency of the encryption algorithm, the relative security of encryption is lower. The definition of security is as follows:

(3) $$\begin{array}{c} s_{k,n}={\left(\frac{f_{k}}{F}\right)}^{2}\frac{1}{u_{k,n}},\;k=1,2,\ldots ,K;n=1,\ldots ,8, \end{array}$$

(4) $$\begin{array}{c} s_{0,n}={\left(\frac{f_{0}}{F}\right)}^{2}\frac{1}{u_{0,n}},\;n=1,\ldots ,8, \end{array}$$

where *s*_*k*,*n*_ represents the security degree of the encryption algorithm *n* executed on the edge server *k* and *s*_0,*n*_ represents the security degree of the encryption algorithm *n* executed on the terminal device.

The edge server can execute eight encryption algorithms, but here it is stipulated that each edge server can execute only one encryption algorithm. Therefore, the choice of each encryption algorithm is defined as a “0-1” variable, and the encryption algorithm selected by the edge server is defined as follows:

(5) $$\begin{array}{c} a_{k,n}=\left\{\begin{array}{c} 0\\ 1 \end{array},\;k=1,2,\ldots ,K;n=1,\ldots ,8\right., \end{array}$$

(6) $$\begin{array}{c} a_{0,n}=\left\{\begin{array}{c} 0\\ 1 \end{array},\;n=1,\ldots ,8\right., \end{array}$$

(7) $$\begin{array}{c} \sum_{n=1}^{8}a_{k,n}=1,\;k=1,2,\ldots ,K, \end{array}$$

(8) $$\begin{array}{c} \sum_{n=1}^{8}a_{0,n}=1, \end{array}$$

where *a*_*k*,*n*_=0 means that the edge server *k* does not execute the encryption algorithm *n* and *a*_*k*,*n*_=1 means that the edge server *k* executes the encryption algorithm *n*. Likewise, *a*_0,*n*_=0 and *a*_0,*n*_=1 represent whether the terminal device implements the encryption algorithm *n*.

The data of the terminal device are offloaded to the edge server for encryption, and the total amount of data needs to be considered. That is, the sum of the encrypted data fragments on the terminal device and the edge server should be equal to the total amount of data waiting for the terminal device. If all the data cannot be encrypted, some unencrypted data will be transmitted in the network in plaintext, which can easily be intercepted by malicious targets and greatly reduce the data security. The constraints on the amount of data here are as follows:

(9) $$\begin{array}{c} m_{0}+\sum_{k=1}^{K}m_{k}=M^{\text{tot}}, \end{array}$$

where *m*_0_ represents the data segment encrypted in the terminal device, *m*_*k*_ represents the data segment encrypted on the edge server *k*, and *M*^*tot*^ represents the total amount of data that the terminal device needs to encrypt.

Because most of the application scenarios of NB-IoT terminal devices are smart meter reading, environmental monitoring, smart door locks, etc., these scenarios usually do not have a continuous power supply, and they can only be powered by batteries. However, because the battery replacement is relatively difficult, once the terminal device is offline from the network due to the exhaustion of capacity, it will have a great impact. Therefore, in order to ensure the continuous working ability of the terminal equipment, the energy consumption of the terminal equipment must be considered in the model. The energy consumption of terminal equipment is mainly generated from two aspects: one is the energy consumed by the terminal equipment when uploading data fragments to the edge server and the other is the energy consumed by the terminal equipment when processing local data fragments. To ensure stable operation of terminal equipment for a long time, it is necessary to limit the energy consumption of terminal equipment. The energy consumption of terminal equipment is defined as follows:

(10) $$\begin{array}{c} \frac{m_{0}}{\sum_{n=1}^{8}a_{0,n}\cdot u_{0,n}}\cdot \beta_{0}+\sum_{k=1}^{K}\frac{m_{k}}{b_{k}}\alpha_{k}\leq E^{\text{local}}. \end{array}$$

The transmit power of the segment *m*_*k*_ is uploaded to the edge server *k*; *b*_*k*_ represents the transmission bandwidth between the terminal device and the edge server *k* and *E*^local^ represents the maximum energy consumption that the terminal device can bear. *m*_0_/∑_*n*=1_^8^*a*_0,*n*_ · *u*_0,*n*_ · *β*_0_ represents the processing energy consumption of the terminal equipment, which is mainly determined by the amount of data to be processed by the terminal equipment, the encryption algorithm executed by the terminal equipment, and the operating power of the terminal equipment. ∑_*k*=1_^*k*^*m*_*k*_/*b*_*k*_*α*_*k*_ represents the transmission energy consumption of the data segment, which is affected by the amount of data transmitted, the transmission bandwidth, and the transmission power.

Similarly, for edge servers, certain energy consumption will be generated when encrypting data fragments uploaded by terminal devices. This part of the energy consumption mainly comes from the processing of data, and each edge server has its own maximum energy consumption limit. Therefore, the energy consumption of the edge server is defined as follows:

(11) $$\begin{array}{c} \frac{m_{k}}{\sum_{n=1}^{8}a_{k,n}\cdot u_{k,n}}\cdot \beta_{k}\leq E_{k},\;k=1,2,\ldots ,K, \end{array}$$

where *E*_*k*_ represents the maximum energy consumption limit that the edge server *k* can bear, *β*_*k*_ is the operating power of the edge server *k*, and *m*_*k*_/∑_*n*=1_^8^*a*_*k*,*n*_ · *u*_*k*,*n*_ represents the data processing time of the edge server *k*, which mainly depends on the amount of data and the encryption algorithm selected by the edge server.

While considering the security of data transmission, the delay should also be taken into account. If the data encryption speed of the edge server is too slow, the performance of the system will also be affected, and the cloud server cannot obtain the data in time. The delay of data transmission is mainly affected by two factors: one is the encryption time of the edge server and the other is the transmission time of the data fragment. Considering the speed of data transmission, it is necessary to limit the delay of data. The delay of data is defined as follows:

(12) $$\begin{array}{c} \max\left\{\max_{k\in K}\left\{\frac{m_{k}}{\sum_{n=1}^{8}a_{k,n}\cdot u_{k,n}}+\frac{m_{k}}{b_{k}}\right\},\frac{m_{0}}{\sum_{n=1}^{8}a_{0,n}\cdot u_{0,n}}\right\}\leq t^{req}, \end{array}$$

where max_*k*∈*K*_{*m*_*k*_/∑_*n*=1_^8^*a*_*k*,*n*_ · *u*_*k*,*n*_+*m*_*k*_/*b*_*k*_} represents the processing time of the data segment by the edge server *k*, which is mainly determined by the transmission time of uploading the data segment to the edge server and the encryption time of the data segment by the edge server. Only when all data fragments are encrypted can the encryption of the whole data be considered complete. Therefore, the time consumed by the edge server that finally completes the encryption is taken as the time consumed by the edge layer to complete the encryption. *m*_0_/∑_*n*=1_^8^*a*_0,*n*_ · *u*_0,*n*_ indicates that the encryption time of the data fragment at the terminal device. *t*^*req*^ is the delay requirement of the cloud server, indicating that the data encryption processing needs to meet a certain delay requirement. The delay of data upload depends on the most time-consuming part of the terminal device and the edge server, and the maximum value should be selected.

The optimization goal of this paper is the overall security of data transmission, and the overall security depends on the data fragments distributed to the edge server and the encryption algorithm selected by the edge server. Among them, the data segment {*m*_*k*_} and the encryption algorithm {*a*_*k*,*n*_} selected by the edge server are used as decision variables. To achieve this goal, the following optimization problem is constructed to maximize the overall security of the data:

(13) $$\begin{array}{c} \text{problem}:S^{ave}=\max\left(\frac{m_{0}}{M^{\text{tot}}}\cdot \sum_{n=1}^{8}a_{0,n}\cdot s_{0,n}+\sum_{k=1}^{K}\left(\frac{m_{k}}{M^{\text{tot}}}\cdot \sum_{n=1}^{8}a_{k,n}\cdot s_{k,n}\right)\right), \end{array}$$

(14) $$\begin{array}{c} \text{subject to}:m_{0}+\sum_{k=1}^{K}m_{k}=M^{\text{tot}}, \end{array}$$

(15) $$\begin{array}{c} \sum_{n=1}^{8}a_{k,n}=1, \end{array}$$

(16) $$\begin{array}{c} \sum_{n=1}^{8}a_{0,n}=1, \end{array}$$

(17) $$\begin{array}{c} \frac{m_{0}}{\sum_{n=1}^{8}a_{0,n}\cdot u_{0,n}}\cdot \beta_{0}+\sum_{k=1}^{K}\frac{m_{k}}{b_{k}}\alpha_{k}\leq E^{\text{local}}, \end{array}$$

(18) $$\begin{array}{c} \frac{m_{k}}{\sum_{n=1}^{8}a_{k,n}\cdot u_{k,n}}\cdot \beta_{k}\leq E_{k}, \end{array}$$

(19) $$\begin{array}{c} \max\left\{\max_{k\in K}\left\{\frac{m_{k}}{\sum_{n=1}^{8}a_{k,n}\cdot u_{k,n}}+\frac{m_{k}}{b_{k}}\right\},\frac{m_{0}}{\sum_{n=1}^{8}a_{0,n}\cdot u_{0,n}}\right\}\leq t^{req}, \end{array}$$

where *m*_*k*_/*M*^*tot*^ · ∑_*n*=1_^8^*a*_*k*,*n*_ · *S*_*k*,*n*_ represents the degree of security obtained after the data segment is encrypted at the edge server *k* and *m*_0_/*M*^*tot*^ · ∑_*n*=1_^8^*a*_0,*n*_ · *s*_0,*n*_ represents the degree of security obtained after encryption by the terminal device. Restriction (14) ensures that all data *M*^tot^ of the terminal device can be encrypted at the edge server. Constraints (15) and (16) indicate that the end device and all edge servers have only one encryption algorithm which is implemented. Constraints (17) and (18) indicate that while considering security, the energy consumption of terminal equipment and all edge servers does not exceed their own energy consumption limits *E*^local^ and *E*_*k*_, which is to ensure that the energy consumption of the equipment is within a certain range. Constraint (19) indicates that the data transmission delay must meet a certain condition *t*^*req*^, which is to maximize the overall security of data transmission and meet the requirement of transmission speed.

The proposed optimization problem is solved hierarchically. By analyzing the problem, it is found that the decision variable {*m*_*k*_} of this optimization problem is a continuous variable, and {*a*_*k*,*n*_} is a “0-1” discrete variable, so the problem is a mixed optimization problem. Moreover, the constraints (14)–(19) couple the two decision variables together, and the solution space increases sharply with the increase of the number of edge servers, so it is very difficult to directly solve the problem with general methods. In order to solve this optimization problem effectively, the original problem needs to be transformed.

The original problem contains discrete optimization part and linear optimization part. Because the two optimization parts are coupled together in the original problem, it is necessary to convert the two parts into a two-layer optimization problem. The idea of layering is to first give the encryption algorithm {*a*_*k*,*n*_} selected by each edge server, and then, the original problem is transformed into the underlying problem, that is, how to optimize the data distribution scheme {*m*_*k*_} when the encryption algorithm {*a*_*k*,*n*_} is given by the edge server. Then, the optimal solution of {*a*_*k*,*n*_} in the top-level problem is obtained by using the data splitting scheme {*m*_*k*_} obtained under the given {*a*_*k*,*n*_}. The bottom problem is a linear optimization problem whose decision variable only contains {*m*_*k*_}, and the top problem is a discrete optimization problem whose decision variable only contains {*a*_*k*,*n*_}.

To effectively solve the optimization problem in the previous section, it is necessary to transform the original problem into multiple subproblems using the idea of stratification. This section stratifies the problem by analyzing the characteristics of the original problem. The layering process is described below.  Figure 2 illustrates the correlation between low-level and top-level issues.

According to the foregoing, given the encryption algorithm $\left\{a_{k,n}\right\}={\hat{a}}_{k,n}\left(k=0,1,\ldots ,K\right)$ of the edge server, the execution efficiency of the encryption algorithm of the server is a known quantity ${\hat{u}}_{k}=\sum_{n=1}^{8}\left({\hat{u}}_{k,n}\cdot {\hat{a}}_{k,n}\right)\left(k=0,1,\ldots ,K\right)$, and the security degree of the server is also a known quantity ${\hat{s}}_{k}=1/{\hat{u}}_{k},\left(k=0,1,\ldots ,K\right)$. Knowing the encryption algorithm, execution efficiency, and security of the edge server, the original problem can be transformed into the underlying problem. Here, the underlying problem can be regarded as the shunting optimization of data {*m*_*k*_}. The underlying problem is as follows:

(20) $$\begin{array}{c} \text{problem}:S^{\text{ave}}=\max\left(\frac{m_{0}}{M^{\text{tot}}}\cdot {\hat{s}}_{0}+\sum_{k=1}^{K}\left(\frac{m_{k}}{M^{\text{tot}}}\cdot {\hat{s}}_{k}\right)\right), \end{array}$$

(21) $$\begin{array}{c} \text{subject to}:m_{0}+\sum_{k=1}^{K}m_{k}=M^{\text{tot}}, \end{array}$$

(22) $$\begin{array}{c} \frac{m_{0}}{{\hat{u}}_{0}}\beta_{0}+\sum_{k=1}^{K}\left(\frac{m_{k}}{b_{k}}\cdot \alpha_{k}\right)\leq E^{\text{local}}, \end{array}$$

(23) $$\begin{array}{c} \frac{m_{k}}{{\hat{u}}_{k}}\beta_{k}\leq E_{k}, \end{array}$$

(24) $$\begin{array}{c} \max\left\{\max_{k\in K}\left\{\frac{m_{k}}{{\hat{u}}_{k}}+\frac{m_{k}}{b_{k}}\right\},\frac{m_{0}}{{\hat{u}}_{0}}\right\}\leq t^{req},\;k=1,2,\ldots ,K, \end{array}$$

Among them, by equivalently transforming the constraints (23) and (24), we can obtain:

(25) $$\begin{array}{c} m_{k}\leq \gamma_{k};\;\gamma_{k}=\min\left\{\frac{E_{k}{\hat{u}}_{k}}{\beta_{k}},t^{req}\cdot {\left(\frac{1}{{\hat{u}}_{k}}+\frac{1}{b_{k}}\right)}^{-1}\right\},\;k=1,2,\ldots ,K, \end{array}$$

(26) $$\begin{array}{c} m_{0}\leq \gamma_{0};\;\gamma_{0}={\hat{u}}_{0}\cdot t^{req}. \end{array}$$

Because 1/*M*^*tot*^ is a constant term in the objective function of the underlying problem, in order to make the problem more concise, omitting this term does not affect the results. At the same time, the following rewrites were made:

(27) $$\begin{array}{c} \frac{\beta_{0}}{{\hat{u}}_{0}}=A_{0}, \end{array}$$

(28) $$\begin{array}{c} \frac{\beta_{k}}{{\hat{u}}_{k}}=A_{k}. \end{array}$$

Bringing formulas (25)–(28) into the underlying problem, the underlying problem can be rewritten as follows:

(29) $$\begin{array}{c} \text{problem}:S^{\text{ave}}=\max\left({\hat{s}}_{0}\cdot m_{0}+\sum_{k=1}^{K}\left({\hat{s}}_{k}\cdot m_{k}\right)\right), \end{array}$$

(30) $$\begin{array}{c} \text{subject to}:m_{0}+\sum_{k=1}^{K}m_{k}=M^{tot}, \end{array}$$

(31) $$\begin{array}{c} A_{0}\cdot m_{0}+\sum_{k=1}^{K}A_{k}\cdot m_{k}\leq E^{\text{local}}, \end{array}$$

(32) $$\begin{array}{c} 0<m_{0}\leq \gamma_{0}, \end{array}$$

(33) $$\begin{array}{c} 0<m_{k}\leq \gamma_{k}, \end{array}$$

(34) $$\begin{array}{c} \gamma_{0}={\hat{u}}_{0}\cdot t^{req}, \end{array}$$

(35) $$\begin{array}{c} \gamma_{k}=\min\left\{\frac{E_{k}{\hat{u}}_{k}}{\beta_{k}},t^{\text{req}}\cdot {\left(\frac{1}{{\hat{u}}_{k}}+\frac{1}{b_{k}}\right)}^{-1}\right\},\;k=1,2,\ldots ,K, \end{array}$$

The underlying problem is solved to obtain a solution $\left\{{\hat{m}}_{k}\right\}\left(k=0,1,\ldots ,K\right)$ about the data segment {*m*_*k*_}, and then according to $\left\{{\hat{m}}_{k}\right\}$, to maximize the overall security *S*^ave^, the optimal solution for the variable {*a*_*k*,*n*_} is obtained. The top-level problem can be viewed as an encryption algorithm selection problem for edge servers:

(36) $$\begin{array}{c} \text{problem}:S^{\text{ave}}=\max\left(\frac{{\hat{m}}_{0}}{M^{\text{tot}}}\cdot \sum_{n=1}^{8}a_{0,n}\cdot s_{0,n}+\sum_{k=1}^{K}\left(\frac{{\hat{m}}_{k}}{M^{tot}}\cdot \sum_{n=1}^{8}a_{k,n}\cdot s_{k,n}\right)\right), \end{array}$$

(37) $$\begin{array}{c} \text{subject to}:\sum_{n=1}^{8}a_{k,n}=1, \end{array}$$

(38) $$\begin{array}{c} \sum_{n=1}^{8}a_{0,n}=1, \end{array}$$

(39) $$\begin{array}{c} \frac{{\hat{m}}_{0}}{u_{0}}\beta_{0}+\sum_{k=1}^{K}\left(\frac{{\hat{m}}_{k}}{b_{k}}\cdot \alpha_{k}\right)\leq E^{\text{local}}, \end{array}$$

(40) $$\begin{array}{c} \frac{{\hat{m}}_{k}}{u_{k}}\beta_{k}\leq E_{k}, \end{array}$$

(41) $$\begin{array}{c} \left.\max_{k\in K}\left\{\frac{\max_{k}\left\{{\hat{m}}_{k}\right\}}{u_{k}}+\frac{{\hat{m}}_{k}}{b_{k}}\right\},\frac{{\hat{m}}_{0}}{u_{0}}\right\}\leq t^{\text{req}},\;k=1,2,\ldots ,K, \end{array}$$

Bringing constraints (30) and (32) into constraints (29), (31), and (33), the underlying problem is transformed into the following equivalent form:

(42) $$\begin{array}{c} \text{problem}:S^{\text{ave}}=\max\left(\sum_{k=1}^{K}\left({\hat{s}}_{k}-{\hat{s}}_{0}\right)\cdot m_{k}+M^{\text{tot}}\cdot {\hat{s}}_{0}\right), \end{array}$$

(43) $$\begin{array}{c} \text{subject to}:A_{0}\cdot \left(M^{\text{tot}}-\sum_{k=1}^{K}m_{k}\right)+\sum_{k=1}^{K}A_{k}\cdot m_{k}\leq E^{\text{local}}, \end{array}$$

(44) $$\begin{array}{c} 0\leq M^{tot}-\sum_{k=1}^{K}m^{k}\leq \gamma^{0}, \end{array}$$

(45) $$\begin{array}{c} 0<m_{k}\leq \gamma_{k},\;k=1,2,\ldots ,K, \end{array}$$

Since $M^{tot}\cdot {\hat{s}}_{0}$ is a constant, omitting it does not affect the result. The above formula can be rewritten as follows:

(46) $$\begin{array}{c} \text{problem}:S^{\text{ave}}=\max\left(\sum_{k=1}^{K}\left({\hat{s}}_{k}-{\hat{s}}_{0}\right)\cdot m_{k}\right), \end{array}$$

(47) $$\begin{array}{c} \text{subject to}:\sum_{k=1}^{K}\left(A_{k}-A_{0}\right)m_{k}\leq E^{\text{local}}-A_{0}\cdot M^{\text{tot}}, \end{array}$$

(48) $$\begin{array}{c} M^{tot}-\gamma_{0}\leq \sum_{k=1}^{K}m_{k},\;\forall k\in K, \end{array}$$

(49) $$\begin{array}{c} \sum_{k=1}^{K}m_{0}\leq M^{tot},\;\forall k\in K, \end{array}$$

(50) $$\begin{array}{c} 0<m_{k}\leq \gamma_{k},\;\forall k\in K, \end{array}$$

## 4. Network Security Technology of Supply Chain Management Based on Internet of Things and Big Data

Supply chain is a network chain structure, which consists of suppliers of core enterprises, suppliers of suppliers, users, and users of users. Generally speaking, the supply chain mainly has the characteristics shown in Figure 3.

The business process and composition of supply chain management are shown in Figure 4. In Figure 4, the manufacturer is the core enterprise, and suppliers and users form a supply chain around the manufacturer to carry out production and operation activities.

As shown in the information model of the node enterprise in the supply chain system in Figure 5, the internal supply chain of the core enterprise carries subsystems, such as production, sales, inventory, finance and procurement, and relevant information. Moreover, core enterprises and upstream suppliers are connected through the Internet to share procurement-related information and carry out supplier relationship management activities. At the same time, core enterprises and downstream sellers or customers also need to share information and carry out business activities according to customer demand information and correct market forecasts.

The EDI-based supply chain information organization and integration model is shown in Figure 6. The settlement center is a value-added network connecting all nodes. After the EDI data information containing all business information is sent to the settlement center, the settlement center will process according to the requirements of different nodes, and after the processing is completed, the relevant documents will be sent back to the relevant nodes.

Secure IoT cloud-to-cloud communication using blockchain is shown in Figure 7. It adds a blockchain-based security layer as a security gateway to the SDN IoT and uses the blockchain as the primary distributed archive.

Due to the device heterogeneity of IoT, there are a large number of resource-constrained devices in the network. These devices can only perform simple sensing, actuation, data processing, etc., functions Moreover, it does not have the ability to carry out higher intelligent forms such as data fusion, and the cost required to achieve a fully distributed Internet of Things is too high to be feasible. Combined with the core idea of edge computing and the main characteristics and security requirements of the Internet of Things, this paper proposes the security architecture of the Internet of Things based on edge computing, as shown in Figure 8.

Based on the above model, the simulation analysis of supply chain nodes is carried out, as shown in Figure 9.

On the basis of the above research, this paper evaluates the network security technology of supply chain management based on the Internet of Things and big data. The security system architecture is constructed through the simulation model, and the simulation attack is carried out on it, the security effect is counted, and the defense effect is counted, and the results are shown in Table 1.

From the simulation data, the network security technology of supply chain management based on the Internet of Things and big data proposed in this paper can realize the effective management and control of supply chain nodes and improve their information security.

## 5. Conclusion

The Internet of Things uses electronic tags and automatic devices in applications, which increases the threat to private data, leads to the disclosure and modification of user information and even malicious tracking and destruction of user data, or leads to the use of private information to do some illegal acts. When using the Internet of Things to process information, the first thing to do is to ensure the integrity and availability of the information. For example, due to network attacks, routing attacks, etc., the data information of the Internet of Things will be incomplete, which will lead to the interruption of Internet of Things applications and the theft of private information. In the application of the Internet of Things, a large number of physical devices in other fields are also required to be connected, which requires the Internet of Things to operate in a stable and reliable environment, so as to ensure the security and integrity of data information during transmission. In order to improve the network security technology of supply chain, this paper studies the Internet of Things and big data technology. From the simulation data, the network security technology of supply chain management based on the Internet of Things and big data proposed in this paper can realize the effective management and control of supply chain nodes and improve their information security.

## Figures and Tables

**Figure 1:** Data offload encryption system model.

**Figure 2:** The relationship between the underlying algorithm and the top-level algorithm.

**Figure 3:** Supply chain structure diagram.

**Figure 4:** Flowchart of supply chain management.

**Figure 5:** Supply chain information model.

**Figure 6:** Supply chain information organization and integration model.

**Figure 7:** Intercloud communication for secure IoT using blockchain.

**Figure 8:** Security architecture based on edge computing and IoT.

**Figure 9:** Simulation diagram of supply chain nodes based on IoT and big data: (a) simulation image 1 of supply chain nodes based on IoT and big data and (b) simulation image 2 of supply chain nodes based on IoT and big data.

**Table 1:** Evaluation of network security technology of supply chain management based on IoT and big data.

No	Security defense	No	Security defense	No	Security defense
1	91.07	19	90.56	37	94.34
2	91.37	20	95.78	38	95.60
3	94.11	21	89.86	39	94.13
4	88.35	22	95.88	40	94.98
5	90.69	23	89.66	41	92.35
6	89.58	24	92.69	42	92.22
7	94.93	25	93.83	43	91.67
8	91.53	26	92.56	44	90.83
9	88.64	27	91.83	45	91.87
10	93.57	28	94.08	46	95.82
11	92.39	29	91.55	47	88.39
12	91.92	30	89.60	48	90.34
13	95.99	31	88.43	49	94.83
14	93.39	32	93.71	50	95.79
15	94.49	33	88.08	51	94.36
16	95.77	34	92.80	52	89.61
17	90.86	35	90.07	53	89.33
18	94.50	36	94.15	54	94.20

## Data Availability

The experimental data used to support the findings of this study are available from the author upon request.
